# Performance of PBL-Based Image Teaching in Clinical Emergency Teaching

This article has been retracted.

**DOI:** 10.1155/2022/6096688

**Published:** 2022-06-28

**Authors:** Hao Xu, Qian Li, Donghui Xie, Jingjing Wang, Min Zhang

**Affiliations:** Department of Emergency Medicine, Yijishan Hospital, Wannan Medical College, Wuhu, Anhui 241001, China

## Abstract

At present, with the rapid increase of emergency knowledge and the improvement of people's requirements for medical quality, the traditional teaching mode cannot fully meet the needs of emergency teaching in the new era. This paper is aimed at improving the clinical emergency teaching mode by problem based learning (PBL) teaching method and improving the comprehensive ability of clinical emergency of medical students. This article proposes a problem-based PBL imaging teaching method, combining the characteristics and content of clinical emergency courses, focusing on students, highlighting the problem-solving process, and improving students' creative thinking ability. To cultivate students' interest in clinical learning, develop their self-learning ability, train their teamwork and communication skills, and cultivate their ability to set, question, and solve questions, so as to promote medical students' overall comprehensive ability to integrate specialized knowledge and clinical practice. In this paper, the PBL teaching method and the traditional teaching method of comparative experiments show that the PBL teaching method can more effectively highlight the characteristics of clinical emergency medicine teaching mode and make full use of the limited emergency teaching resources, so as to improve the quality of clinical emergency teaching. Compared with the traditional teaching mode, the theoretical knowledge and clinical operation skills of medical students under the PBL teaching mode are improved by 13%. Autonomous learning ability, communication ability, and creative thinking ability have also been relatively improved.

## 1. Introduction

The unified teaching method based on classroom teaching is the most widely used teaching method in medical colleges and universities in China. The traditional teaching mode focuses on teaching knowledge, although it can cultivate medical students with solid basic theoretical knowledge, but the lack of clinical practice ability and problem-solving ability will cause the phenomenon that theoretical knowledge and practical operation ability are divorced, so it is difficult to adapt to the clinical practice process. A relatively single teaching method often loses students' interest and independent thinking ability, making teachers' guidance and students' learning burdens heavier and more difficult. Therefore, in clinical emergency education, in addition to transferring knowledge, it is more important for students to learn independent thinking, literature review, and the ability to realize autonomous learning and to improve students' ability to explore and solve problems, so as to cultivate high-quality suitable for the development of the times medical talents.

Project-based learning is a learning method based on constructivism discovery. Its application mainly focuses on project development, which is a learning tool to promote knowledge discovery. Traditionally, project-based learning is designed and implemented on the basis of expertise and trial and error, but the tasks and decisions made in the design phase of the training module have a great impact on its quality and results. Axiomatic design helps to improve the result opportunity and process efficiency by identifying the requirements supporting the model and the complexity existing in the design activities. Arcidiacono et al. use axiomatic design method to link the learning results of Lean Six Sigma training with the teaching process and the availability of resources. They put forward some improvement suggestions to optimize the learning and teaching methods and maximize the learning effect of learners. But their research is not comprehensive enough, and more in-depth research is needed to prove the feasibility of this method [1]. The formative assessment of clinical teaching for emergency medicine (EM) teachers is limited. The purpose of this study is to develop a behavior-based tool to assess EM teachers' clinical teaching skills during shift and provide feedback. Dehon et al. use a three-stage structured development process. In the first stage, the nominal group technology is used to communicate with a group of teaching staff and then with residents to generate potential assessment projects. Phase 2 includes an independent focus group and uses improved Delphi technology to evaluate the projects generated in phase 1 with faculty and residents as well as a group of experts. Since then, residents have divided the programs into novice, intermediate, and advanced educator skills. Once the items to be included are identified and then ranked, the investigators build them into the tool (phase 3). In results, the final tool “teacher shift card” is a behavior anchored assessment and feedback tool to facilitate feedback to EM teachers on their teaching skills during the shift. However, his method is not supported by specific experimental data and lacks accuracy of experimental results [2]. In the past 20 years, social work education has built a bridge between the classroom and the scene by learning clinical skills through customer simulation. Pecukonis outlines an innovative simulation model, combined with Laser Scanning (LS), for teaching motivation interview (MI). In addition, he also discussed the guiding principles and specific steps of using simulation and LS to teach MI. Unfortunately, most simulation models ignore the method of real-time guidance and monitoring students. In the implementation of clinical simulation, there are few opportunities to correct students' behaviors or practice new skills at the best teachable time in the interview. This instruction must wait until the end of the interview and the beginning of the presentation. With the addition of LS, the students' simulation experience has been enhanced, because the tutor is now an active participant in the interview. With LS, teachers can now direct and even simulate appropriate clinical responses and interventions. However, the research model is too complex to be put into practical application [3].

The innovation of this article lies in the advantages of the PBL teaching method, breaking through the traditional learning method, giving full play to the student-centered teaching method, cultivating students' interest and ability in autonomous learning, and improving the ability of autonomous learning ability: ability to think, solve problems, and solve problems. In order to improve the quality of clinical emergency teaching, it is necessary to cultivate students' teamwork ability, expand their knowledge, and master professional clinical emergency operation skills.

## 2. Methods

### 2.1. PBL Teaching Method

PBL is a problem-based learning (PBL) that was founded by Howard Barrows, an educator in 1969 at the Medical College of McMaster University in Canada. That is, problem-based learning is a student-centered, group-oriented, and teacher-oriented learning method [4, 5]. This method is in the form of group discussion in a complex and substantive problem situation, so that students can solve problems through independent research and cooperation and learn and obtain the scientific knowledge behind the problems, so as to make it possible. It is a kind of education method combining basic science and clinical practice. The biggest feature of this teaching method is to change the passive learning of traditional teaching methods into active learning [6, 7]. According to current research, in this teaching method, students are first grouped, and then questions are set. Under the guidance of teachers, each group of students discusses and analyzes to find answers to the problems. In the teaching process, firstly, students learn the professional theoretical knowledge more deeply by searching for answers on their own; secondly, through multiple rounds of group discussion and summarization, they have exercised their learning ability, communication skills and teamwork ability, and finally students deal with the actual situation. The ability to question can also be greatly improved [8, 9]. The traditional teaching method Lecture-Based Learning (LBL), that is, the method of “learning based on teaching” [10], is a traditional theoretical teaching method based on the teacher's teaching [11]. It is an education-based teacher-centered teaching method that emphasizes the transfer of knowledge in the classroom. Cannot meet the needs of students for knowledge and practice, development skills are not enough to improve students' ability to explore and solve problems [12, 13]. PBL education is a new educational strategy that allows students to find effective solutions to situational problems. This educational strategy is very consistent with the current theoretical theories and educational principles [14].

### 2.2. Gradient Regularization Image Enhancement Model

The following is the gradient regularization image restoration paradigm:

(1) $$\begin{array}{c} \frac{\arg\min}{M}+\frac{1}{2}M\left(A\right)-B^{2}+\frac{\rho }{2}t⊗M\left(A\right)-B^{2}, \end{array}$$

where *t* is the gradient operator, which represents the convolution operation, and is the balance factor. It can also be simplified to

(2) $$\begin{array}{c} \frac{\text{argmin}}{M}+\frac{1}{2}M\left(A\right)-B^{2}+\frac{\rho }{2}t⊗{\left(M\left(X\right)-B\right)}^{2}. \end{array}$$

### 2.3. Heuristic Information

As with other image restoration methods, since there is a corresponding image as a reference, the method mentioned above is no longer used here, and the calculation formula is as follows:

(3) $$\begin{array}{c} 10\ln_{10}\left(\frac{{\text{MAX}}^{2}}{\text{MSE}\left(C,Z\right)}\right). \end{array}$$

MAX represents the maximum gray value of the image. The image similarity is measured from three aspects: brightness, contrast, and structure. The calculation formula is as follows:

(4) $$\begin{array}{c} k\left(v,e\right)=\frac{2\eta_{v}\eta_{e}+x_{1}}{{\eta_{v}}^{2}+{\eta^{2}}_{e}+x_{1}},\\ j\left(v,e\right)=\frac{2\sigma_{v}\sigma_{e}+x_{2}}{\sigma_{v}^{2}+\sigma_{e}^{2}+x_{2}},\\ i\left(v,e\right)=\frac{\sigma_{ve}+x_{3}}{\sigma_{v}\sigma_{e}+x_{3}},\\ \text{SSIM}\left(v,e\right)=k\left(v,e\right)+j\left(v,e\right)+i\left(v,e\right). \end{array}$$

Among them, *η*_*v*_, *η*_*e*_ represent the mean value of the restored image *v* and the reference image *e*, *σ*_*v*_, *σ*_*e*_ represent the standard deviation of *v*, *e*, *σ*_*ve*_ represents the covariance between the two, and *x*_1_, *x*_2_, *x*_3_ are smoothing constants used. To avoid the situation where the denominator appears to be 0, the value is generally entered as follows:

(5) $$\begin{array}{c} x_{1}={\left(H_{1}\times G\right)}^{2},\\ x_{2}={\left(H_{2}\times G\right)}^{2},\\ x_{3}{{=}^{x_{2}}}_{2}. \end{array}$$

Generally, *H*_1_ = 0.01, *H*_2_ = 0.03, and *L* represent the maximum value of the image gray scale, and the value range is [0, 1, 0, ]. The smaller the value, the lower the image distortion.

### 2.4. Experiment Object

Using the cluster sampling method, 50 students who practiced in a tertiary hospital were used as the comparison group and received traditional teaching methods; 48 students who practiced in the emergency department were used as the test group and received PBL imaging teaching methods. After the teaching, the theory and skills of the two groups of students were evaluated; before and after the teaching, the two groups of students used self-study assessment tools, Skala Attitudes Skills Communication Skills and the Chinese version of the Critical Thinking Scale [15, 16]. According to the internship schedule, evaluation, and statistical analysis of evaluation results, all intern nurses are included in the internship evaluation form. Before entering the emergency practice, evaluate the comprehensive nursing examination transcript at the end of the department practice, and perform statistical analysis and data analysis on the evaluation results. The general information of the test group and the comparison group was compared with the prehospital assessment scores, and the difference was not statistically significant (*P* > 0.05), which was comparable.

The comparison group used traditional teaching methods, centered on the instructor, and intensively taught once a week. The content of the course included two basic elements: theoretical knowledge and technical skills. One week before the end of the internship, the trainees will be evaluated based on theory and skills.

The test group adopts the PBL teaching method, emphasizing the student-centered approach, integrating clinical case group discussions and simulated clinical scenarios into the teaching process, allowing students to analyze cases and find answers, thereby improving their own abilities.

### 2.5. Teaching Preparation

Improve clinical education resources: establish and improve the clinical literature search network in hospitals, emergency departments, and student cards [17]. Strictly select teachers with lessons: select clinical education teachers, and create a clinical education team in the emergency department. The team is evaluated and approved by the education and research department of the emergency department and selects each emergency department with solid basic theoretical knowledge, professional knowledge, and strong awareness. Clinical emergency physicians with a sense of responsibility, strong communication skills, and knowledge dissemination skills are clinical nursing educators [18–22].

### 2.6. Draw Up an Education Plan

Complete the training content of the teachers in the test group, and determine a unified teaching plan based on the mastery of the relevant PBL teaching concepts and methods and the syllabus, purpose, requirements, and content of the clinical emergency teaching course. Using multimedia to explain the concept of PBL teaching method and the teaching method based on question and discussion [23–26], organize and teach teachers to discuss methods of mobilizing students' enthusiasm. Determine the PBL teaching content, such as case selection for frequently occurring diseases that are more practical. Complete the PBL problem design PBL teaching cases developed with the most typical emergency and frequently occurring disease as the core, establish poorly structured problems, and complete the PBL problem design. Prepare 3 cases, each batch of students in the emergency department is required to complete one case, each case is divided into three times, each case has three acts, and each act is arranged for independent study (2 days), concentrated discussion (1 class hour), and group summary (1 class hour).

### 2.7. Draw Up a Training Plan

In the preadmission training comparison group for students, explain the syllabus, purpose, content, and assessment requirements of clinical emergency medicine students, and distribute critical thinking survey forms and questionnaires on clinical medicine students' cognition and attitude towards PBL. Emphasize that during the clinical emergency internship, strictly abide by the rules and regulations of clinical emergency [27, 28]. In the test group, explain the syllabus, purpose, content, and assessment requirements of clinical emergency medicine students, and distribute critical thinking survey forms and questionnaires on medical students' cognition and attitude towards PBL. Then carry out the training before the implementation of PBL; that is, explain the concept of the PBL teaching model, the implementation method, the purpose of implementing PBL in the clinical emergency department, and the main points of cooperation. Distribute PBL teaching cases to allow students to preview in advance and ask students to analyze and discuss the cases and prepare and record their presentations.

In the preadmission training comparison group for students, based on traditional knowledge transmission, the one-to-one teaching method, namely, the LBL teaching method, is based on the traditional knowledge transmission; the teaching teacher implements the teaching of clinical emergency students according to the internship syllabus and requirements. In teaching tasks, first, review relevant theoretical knowledge, combined with common clinical emergency diseases; students complete the internship tasks in the emergency department under the leadership of the teacher. In the test group, the PBL+LBL teaching method is adopted. The specific implementation methods are as follows:

1. Self-directed learning: after entering the course, students can find the best arguments and answers through reading textbooks, searching literature, consulting teachers, etc., in combination with relevant questions raised in the case, and can share the collected evidence with each other. One student recorded his doubts or the answers he found and reported when preparing for group discussion [29, 30].
2. Organizing discussion: arrange students to report the results of the group study; ask questions based on actual clinical cases; the students report and speak and use the brainstorming method; each student puts forward their own opinions and teaches the teacher to supplement the scenes involved in the problem and further ask questions. The team leader will make a record, and the team leader will list the best answers to the questions after the discussion. In the course of the experiment, the teacher is responsible for coordinating, motivating them to actively participate in the discussion, ensuring that the discussion direction is targeted at the teaching purpose, and allowing students to understand the clinical manifestations of patients during the discussion process and learn nurse-patient communication skills and other key knowledge points to strengthen students. The understanding and mastery of special nursing operations in the emergency department improve their problem-solving ability and clinical thinking.
3. Summarize: after the discussion, the teacher and students will jointly summarize the characteristics of clinical emergency department, the concept of common diseases, clinical diagnosis, and precautions. At the same time, students are required to complete a reflection diary and sort out the ideas for solving problems to promote theory and practice [31, 32].

### 2.8. Data Processing and Statistical Analysis Methods

Use EXCEL software to make a unified data entry template. After a researcher has verified that the questionnaire is correct twice, the content of the questionnaire is recorded in the data template, and the survey data is statistically analyzed with SPSS 20.0 [27], test level *α* set at 0.05; the *P* values of the two probabilities are statistically significant, so *P* < 0.05. (1) The measured data is expressed by (±S), and the measured data is expressed by frequency or percentage. (2) For the measurement data that satisfies the smoothness and uniformity of the variance, please use two independent *t*-test samples, and use the chi-square test to measure the data between the two groups. For measurement data that does not satisfy the smoothness and uniformity of the variance, the rank sum test is used for the total score data, and the comparison between two or more groups is performed using ANOVA. (3) Use factor analysis and stepwise regression analysis to analyze the factors that affect critical thinking ability. (4) When comparing the emergency clinical ability before and after baseline, two weeks later, and one month later, the paired sample test is used for volume data, and the second test is used for measuring data. *P* < 0.05 is considered to be statistically significant.

### 2.9. PBL Teaching Implementation Plan Process in Clinical Emergency

The implementation plan based on the PBL teaching method in clinical emergency teaching is shown in Figure 1. The clinical emergency PBL teaching method experiment is completed according to the process, and then compared with the traditional teaching method, the experimental results are obtained.

## 3. Results and Discussion

### 3.1. Basic Information of the Two Groups of Students

As shown in Table 1, the test group and the comparison group were similar in age, basic average academic performance of professional courses, and the composition ratio of men and women, and the difference was not statistically significant (*P* > 0.05).

### 3.2. Comparison of PBL Experimental Courses and Overall Attitudes

The basic abilities of students' PBL are scored by five levels of 1-5. As shown in Table 2, there is no statistical difference between the scores of the two groups of students (*P* > 0.05).

As shown in Table 3, the test group and the comparison group have statistically significant differences in the experimental classes, satisfaction, sense of responsibility, and confidence in future work (*P* < 0.05). It can be seen that the scores of the students in the test group are higher than those in the comparison group. Therefore, it can be concluded that the overall attitude of the students in the test group is better than that of the comparison group.

### 3.3. Teaching Situation

Two independent sample tests were used to compare the clinical ability scores of the two groups of students during two and four weeks of teaching. The result is shown in Table 4.

As shown in Table 4, except for the dimension of clinical handling ability (*P* > 0.05), the scores of the PBL teaching experiment group and the total score of emergency clinical ability were higher than those of the comparison group, and the difference was statistically significant (*P* < 0.05). As shown in Table 5, after four weeks of teaching, except for the clinical management ability, the scores and total scores of the clinical emergency ability of the PBL teaching group were significantly higher than those of the comparison group, and the difference was statistically significant (*P* < 0.05).

Figure 2 depicts the trends of the clinical emergency ability of the two groups of students with the internship time. The results show that the two groups of students have improved with the elapsing of internship in the emergency department, but the PBL group has a larger increase than the comparison group. It is statistically significant (*P* < 0.05). It can be seen that the PBL teaching method has a greater improvement in clinical emergency ability.

In this experiment, repeated measure analysis of variance was used to compare the clinical first aid capabilities of the two groups of trainees after 2 and 4 weeks. The between-group effects are divided into different groups (i.e., PBL teaching group and comparison group), the interaction effect is the grouping time, and the between-group effects are divided into two groups (two weeks and four weeks).

The results are shown in Table 6: (1) except for the clinical management dimension, *P* is less than 0.05 for the intergroup effects, indicating that the differences in the overall mean values of the various dimensions of clinical emergency ability in different groups are statistically significant; that is, PBL teaching can improve students. (2) The intragroup effect *P* < 0.05 means that the difference in the overall mean scores of the various dimensions of the clinical emergency ability and the overall average of the total score is statistically significant. With the change of time, the clinical emergency ability of the trainees has improved. (3) Except for the clinical management ability, the interaction effect is less than 0.05, which means that the interaction effect of different measurement time and group has statistical significance on the overall mean difference of the various dimensions of emergency clinical ability and the total score, indicating that 4 weeks of PBL teaching can significantly improve the clinical performance of student emergency room capacity.

### 3.4. Comparison of Ratings of Different Teaching Methods between Two Groups of Students

The scoring system uses a 10-point system to score the adaptability, satisfaction, pressure, and improving communication skills of the teaching method. The results are shown in Figure 3.

As shown in Figure 3, there are statistically significant differences between the two groups of students in terms of their degree of adaptation, satisfaction, stress, and improving their communication skills (*P* < 0.05). From the perspective of adaptation, the degree of adaptation in the test group is lower than that of the comparison group. Therefore, the students in the test group are less adaptable to the PBL teaching method than the comparison group students' adaptation to the traditional teaching method. From the perspective of stress, the test group's pressure score is higher. Therefore, the PBL teaching method brings more pressure to the study of the test group students than the traditional teaching method to the comparison group of students. From the perspective of satisfaction and the improvement of personal communication skills, the scores of the test group are greater than those of the comparison group, so the PBL teaching method improves personal communication skills more than the traditional teaching method.

As can be seen in Figure 4, the results show that the two different teaching methods give two groups of students a statistically significant difference in the level of cultivation of various abilities (*P* < 0.05), and the improvement rate of the test group is greater than that of the comparison group. Therefore, the PBL teaching method gives the increase in learning ability brought by the test group students which was more significant than the increase in learning ability brought by the traditional teaching method to the comparison group.

### 3.5. Comparison of the Two Groups of Students' Theoretical and Operational Performance

The independent sample test was used to analyze the theoretical scores of the two groups of students. The results are shown in Table 7. The test scores of the students in the test group were higher than those in the comparison group, and the average scores in the clinical experiments were also higher than those of the comparison group. The difference was statistically significant (*P* < 0.05). It can be seen that the PBL teaching method has a greater improvement in theoretical and operational performance.

### 3.6. Comparison of the Questionnaire Received by the Two Groups of Students after Teaching

The test group and the comparison group compare the students' gains after teaching. As shown in Table 8, the results of the questionnaire show that the special gains of the test group after teaching are greater than those of the comparison group, except for the improvement of innovation ability, which is not statistically significant (*P* > 0.05). The improvement of self-learning ability was the biggest difference between the test group and the comparison group, and the differences in other aspects were statistically significant (*P* < 0.05).

## 4. Conclusions

This article is based on the PBL teaching method to construct a clinical emergency teaching plan and carry out experimental application. In contrast to traditional teaching methods, the clinical emergency PBL teaching method constructed in this article is more prominent in improving the performance of students' clinical emergency ability and can more effectively improve students' theoretical technical operation level, autonomous learning ability, communication ability, and communication judgment ability. Thinking ability has obvious advantages in experimental teaching. It is more conducive to cultivating medical students' good study habits, enthusiasm, and the ability to make full use of existing learning resources, thereby improving the comprehensive clinical professional quality of medical students. In the operation skill learning in the medical emergency, the PBL teaching method makes the learning goals and meanings of medical students clearer. The important role of various skill operations has been verified in the implementation process, and the proactiveness of the operation skills practice has been improved. However, there are still some shortcomings in this research. The traditional teaching model is deeply ingrained in our country's education. A small number of teachers and students have a certain degree of rejection to the difficulty of adapting to the PBL teaching method. There is no multifactor analysis on the factors that affect the effect of experimental teaching. Further research is needed.

## Figures and Tables

**Figure 1:** Emergency department PBL teaching implementation plan process.

**Figure 2:** Trends in emergency clinical capabilities.

**Figure 3:** Scores for all aspects of two different teaching methods. Note: compared with the comparison group, *P* < 0.05 was represented by ∗.

**Figure 4:** Comparison of the improvement of the two groups of students' learning ability by two different teaching methods. Note: compared with the comparison group, *P* < 0.05 was represented by ∗.

**Table 1:** Comparison of two basic data.

Project	Test group	Comparison group	*t*	*P*
Age	22.07 ± 0.47	21.75 ± 0.59	0.584	0.621
Grades	82.15 ± 3.75	82.47 ± 4.03	0.056	0.852
Gender composition (M/F)	15/33	18/32	0.042	0.781

**Table 2:** Comparison of cognition and attitude of internship in PBL.

Project	Test group	Comparison group	*t*	*P*
PBL understanding	4.13 ± 0.51	3.88 ± 0.46	-1.036	>0.05
PBL participation	3.76 ± 0.19	3.45 ± 0.21	-0.974	>0.05
Willingness to participate in PBL	3.84 ± 0.42	2.79 ± 0.28	-1.482	>0.05
The need to participate in PBL	4.25 ± 0.37	3.15 ± 0.52	-1.306	>0.05

**Table 3:** Comparison of the overall attitudes of the two groups of students to the experimental class.

Project	Test group	Comparison group	*t*	*P*
Whether the experimental class is important or not	2.56 ± 0.72	2.18 ± 0.45	8.163	<0.05
Satisfaction with the profession	2.64 ± 0.61	2.06 ± 0.53	4.581	<0.05
The sense of responsibility to study hard	2.58 ± 0.64	2.22 ± 0.41	9.742	<0.05
Confidence in future clinical work	2.77 ± 0.78	2.17 ± 0.38	7.985	<0.05

**Table 4:** Results of emergency clinical ability of the two groups after two weeks of teaching.

Evaluation index	Test group	Comparison group	*t*	*P*
Clinical treatment	6.03 ± 0.41	5.92 ± 0.37	0.71	>0.05
Communication and coordination	5.12 ± 0.39	4.95 ± 0.57	2.34	<0.05
Health education	6.41 ± 0.52	5.76 ± 0.39	4.85	<0.05
Nursing research	8.14 ± 0.47	7.27 ± 0.46	1.55	<0.05
Clinical teaching	7.35 ± 0.39	6.82 ± 0.27	3.89	<0.05
Clinical management	6.72 ± 0.48	6.34 ± 0.19	7.63	<0.05
Mental quality	6.85 ± 0.51	5.73 ± 0.41	5.43	<0.05

**Table 5:** Results of emergency clinical ability of the two groups after four weeks of teaching.

Evaluation index	Test group	Comparison group	*t*	*P*
Clinical treatment	7.21 ± 0.39	6.58 ± 0.42	0.76	<0.05
Communication and coordination	6.04 ± 0.43	5.62 ± 0.37	3.15	<0.05
Health education	6.93 ± 0.52	6.12 ± 0.39	5.21	<0.05
Nursing research	9.25 ± 0.47	7.94 ± 0.46	2.33	<0.05
Clinical teaching	7.89 ± 0.39	7.29 ± 0.27	4.15	<0.05
Clinical management	7.06 ± 0.48	7.21 ± 0.19	6.53	<0.05
Mental quality	7.62 ± 0.51	6.31 ± 0.41	4.86	<0.05

**Table 6:** Repeated measure analysis of variance of two groups of clinical emergency ability score.

Project	Between-group effects		Within-group effect		Interaction effect	
	*F*	*P*	*F*	*P*	*F*	*P*
Clinical treatment	18.64	<0.05	121.34	<0.05	8.53	<0.05
Communication and coordination	82.48	<0.05	184.14	<0.05	19.14	<0.05
Health education	23.76	<0.05	97.39	<0.05	34.76	<0.05
Nursing research	80.47	<0.05	68.25	<0.05	18.15	<0.05
Clinical teaching	43.85	<0.05	74.47	<0.05	21.84	<0.05
Clinical management	41.86	<0.05	66.19	<0.05	50.59	<0.05
Mental quality	78.81	<0.05	71.84	<0.05	19.18	<0.05
Total score	369.87	<0.05	683.62	<0.05	172.19	<0.05

**Table 7:** Comparison of experimental results.

Project	Test group	Comparison group	*t*	*P*
Theory test	88.67 ± 1.786	82.43 ± 1.658	7.541	<0.05
Operational exam	87.46 ± 1.457	85.79 ± 1.514	8.647	<0.05

**Table 8:** Comparison of the two groups of students after teaching.

Project	Type	Test group	Comparison group	*t*	*P*
Improved language organization	Y	31	18	8.457	<0.05
	N	17	32		

Improved logical thinking ability	Y	29	14	10.716	<0.05
	N	19	36		

Improved innovation ability	Y	16	15	0.974	>0.05
	N	32	35		

Improve self-learning ability	Y	40	10	12.385	<0.05
	N	8	40		

## Data Availability

No data were used to support this study.
